The article "Application of Da Vinci Robot and Thoracoscopy in Radical Lung Cancer Surgery" was retracted in 2023. Reasons: unreliable results or conclusions; lack of ethics approval or compliance; concerns about the data; concerns about the peer review.

# Application of Da Vinci Robot and Thoracoscopy in Radical Lung Cancer Surgery

**DOI:** 10.1155/2022/2011062

**Published:** 2022-03-16

**Authors:** Fenqiang Qi, Minfeng Xiang, Yuxin Deng, Wei Huang, Yan Sun

**Affiliations:** ^1^Department of Cardiothoracic Surgery, Liuzhou Workers Hospital, The Fourth Affiliated Hospital of Guangxi Medical University, Liuzhou 545007, China; ^2^Department of Scientific Research, Liuzhou Workers Hospital, The Fourth Affiliated Hospital of Guangxi Medical University, Liuzhou 545007, China

## Abstract

In this article, we have explored the feasibility and safety of Da Vinci's robotic surgery system in the radical resection of lung cancer. For this purpose, 73 cases of patients with lung cancer who underwent radical resection in the thoracic surgery of our hospital, particularly from July to September 2020, were collected, of which 22 cases operated with the Da Vinci robot were the Da Vinci robot group, including 11 men and 11 women. The 51 patients who underwent thoracoscopic surgery were in the thoracoscopic group, including 24 males and 27 females. All 22 patients in the Da Vinci robot group completed the operation under the Da Vinci robot operation system without conversion to thoracotomy. In the thoracoscopic group, 49 patients successfully completed the operation under thoracoscopy, and 2 patients were converted to thoracotomy. There was a significant difference between the two groups in the average operation time and the number of lymph nodes, but there was no significant difference in the amount of intraoperative bleeding and postoperative hospital stay. Compared with thoracoscopic radical lung cancer surgery, Da Vinci's robotic surgery system is equally safe and effective, and more lymph nodes are cleaned during surgery.

## 1. Introduction

With the development of imaging technology and the popularization of routine physical examination, lung cancer patients are found more and more early [1, 2]. According to statistics, the incidence rate and mortality rate of lung cancer in China are the first [3] of all malignancies. The incidence rate and mortality rate of men are the highest. In women, the incidence rate has jumped to second place, only after breast cancer, and its mortality rate has ranked first in [4]. Moreover, the incidence rate of women is higher than that of male [5] worldwide. China has made great progress in the treatment of lung cancer in recent years. It has a variety of treatment methods, including surgical treatment, chemotherapy, radiotherapy, and molecular targeted therapy with major breakthroughs in the latest research [6], which have achieved good therapeutic effects. However, so far, early surgical treatment of lung cancer is still the only way to cure lung cancer. Thoracotomy is traditionally used, but with the improvement of surgical technology and the continuous development of minimally invasive surgery, thoracoscopic radical resection of lung cancer in many domestic hospitals has gradually replaced thoracotomy and become a conventional surgical method for the treatment of lung cancer, and its safety and effectiveness have been widely affirmed [7–10]. Through years of practice, thoracoscopy technology has been widely used and developed in China [9, 11, 12]. NCCN (National Comprehensive Cancer Network) guidelines recommend thoracoscopy as the preferred surgical method for radical resection of lung cancer. However, due to the limitations of thoracoscopy and its surgical instruments, there will be a certain blind area in the operation, and the instrument arm is long, straight, and hard, which makes it difficult to carry out more complex thoracoscopic surgery. With the continuous development of endoscopic technology, minimally invasive surgery has become the trend of surgical development in the future [13]. The advent of Da Vinci's robot surgery system has promoted the further development of minimally invasive surgery. In 2001, Yoshino and others took the lead in thoracic surgery and successfully performed thymectomy for a 74-year-old male patient [14]. However, the wide application of the Da Vinci surgical system in thoracic surgery is relatively late, which may be related to the high risk of intrathoracic surgery, the relative concentration of important organs, nerves, and major blood vessels in the thoracic cavity, difficult operation, easy accidental injury, and other reasons [15]. At present, the fourth generation Da Vinci's robotic surgery system developed by innovative surgical has been widely used in the clinic. The birth and development of Da Vinci's robotic surgery system have further promoted the development of minimally invasive surgery, which also indicates the advent of the third generation surgery era and will lead the new direction of minimally invasive surgery in the future [16]. The purpose of this study is to analyze and compare the perioperative treatment effects of Da Vinci's robotic surgery system and thoracoscopy in radical resection of lung cancer. By collecting clinical cases, analyzing clinical statistical data, and comparing the data differences, we can explore whether the application of Da Vinci's robotic surgery system in radical resection of lung cancer is as safe and effective as thoracoscopy or even better than thoracoscopy.

The article "Application of Da Vinci Robot and Thoracoscopy in Radical Lung Cancer Surgery" was retracted in 2023. Reasons: unreliable results or conclusions; lack of ethics approval or compliance; concerns about the data; concerns about the peer review.

### 1.1. Da Vinci

Compared with traditional thoracoscopy, the fourth generation Da Vinci robot can clearly present the dense blood vessels and trachea in the lungs, and the intricate threads between diseased tissues and normal tissues in front of the surgeon, so that the doctor can be more clear and more intuitively distinguish the diseased tissue. At the same time, it can also filter out the slight tremor of the operator's hand during operation.

Figure 1 shows the Da Vinci fourth generation equipment.

In terms of lymph node dissection, the Da Vinci robot also has excellent performance. The surgical field with almost no dead corner can more clearly expose the lymph nodes in the hilar and mediastinal regions, greatly reduce the incidence of residual lymph nodes, and avoid the damage to normal nerves and blood vessels to the greatest extent.

In this article, we have explored the feasibility and safety of Da Vinci's robotic surgery system in the radical resection of lung cancer. For this purpose, 73 cases of patients with lung cancer who underwent radical resection in the thoracic surgery of our hospital, particularly from July to September 2020, were collected, of which 22 cases operated with the Da Vinci robot were the Da Vinci robot group, including 11 men and 11 women. The 51 patients who underwent thoracoscopic surgery were in the thoracoscopic group, including 24 males and 27 females. All 22 patients in the Da Vinci robot group completed the operation under the Da Vinci robot operation system without conversion to thoracotomy.

The remaining paper is organized as follows.

In section 2, data and equipment which are utilized in this study are described in detail.

## 2. Data and Equipment

### 2.1. Clinical Case Data

Among them, 22 patients underwent surgery with the Da Vinci robot and were classified into the Da Vinci robot group. There were 11 males and 11 females, aged 39–78 years, with an average age of (60.7 ± 8.2) years. 51 patients underwent thoracoscopic surgery. They were divided into the thoracoscopic group, 24 males and 27 females, aged 43–82 years, with an average of (59.0 ± 9.5) years. According to the postoperative pathological report, there were 15 cases of adenocarcinoma, 4 cases of squamous cell carcinoma, 2 cases of adenosquamous cell carcinoma, and 1 case of large cell carcinoma in the robot group. In the thoracoscopy group, there were 33 cases of adenocarcinoma, 12 cases of squamous cell carcinoma, 1 case of adenosquamous cell carcinoma, 3 cases of large cell carcinoma, and 2 other cases. Preoperative chest enhanced CT showed pulmonary space-occupying lesions in both groups. The preoperative examination was improved, and there was no distant metastasis, suggesting that the mass can be cut. All patients were treated with inhalation and intravenous anesthesia, double-lumen endotracheal intubation, and contralateral one lung ventilation.

The article "Application of Da Vinci Robot and Thoracoscopy in Radical Lung Cancer Surgery" was retracted in 2023. Reasons: unreliable results or conclusions; lack of ethics approval or compliance; concerns about the data; concerns about the peer review.

### 2.2. Da Vinci's Robotic Surgery System

Da Vinci's robotic surgery system is mainly composed of three parts, namely, the surgeon's operation control system, the bedside manipulator operation system, and the high-definition imaging display system. The effect is shown in Figure 2.

#### 2.2.1. Operation System of Chief Surgeon

The chief surgeon operates the handle ring by watching the 3D image of the 3D display system on the console, and his feet can complete a series of operations such as electrocoagulation and electric cutting through the foot pedal. Moreover, the surgeon's surgical field of vision is a 3D image with strong stereoscopic sense, and the image can be enlarged by 10 times. In such a high-definition surgical field of vision environment, it can easily identify various tissue structures, carry out more detailed surgical operations, and avoid accidental injury to nerves and blood vessels.

#### 2.2.2. Bedside Manipulator Operating System

The bedside operating system of Da Vinci's robotic surgery system is composed of a mirror-holding arm, a working arm, an endoscope, and surgical instruments connecting the mirror-holding arm and the working arm. Generally, there is only 1 mirror-holding arm and 2-3 operating arms. The operating arm can imitate the action of the human hand, and its mobility is higher than that of the human hand joint, and the rotatable angle is larger. It can complete the fine operation that the human hand cannot complete in the narrow operating space [17]. Compared with human hands, the mechanical arm of the Da Vinci robot has another advantage; that is, it can automatically filter out the trembling action of human hands through computer processing and automatically reduce the excessive operation range of the chief surgeon, making it more precise and stable [18].

#### 2.2.3. High-Definition Imaging Display System

The traditional thoracoscopy is two-dimensional imaging, so that the surgeon cannot well identify the spatial and three-dimensional position relationship between tissues. The 3D imaging technology of Da Vinci's robotic surgery system can completely display the spatial position relationship of various tissue structures and can freely enlarge or narrow the surgical field of vision according to different tissue positions and the personal visual habits of the surgeon.

## 3. Proposed Method

### 3.1. Data Acquisition

#### 3.1.1. Clinical Case Data Collection

Lung cancer cases were retrieved through the case management system of our hospital. The search conditions include that between July and September 2020, Da Vinci robot assisted radical resection of lung cancer and thoracoscopic radical resection of lung cancer. According to the following inclusion criteria and exclusion criteria, a total of patients who underwent surgery with the Da Vinci robot were collected and classified into the Da Vinci robot group.

1. Postoperative pathological report confirmed lung cancer
2. The TNM stage of lung cancer is stage I A—III B
3. The operation method was the Da Vinci robot-assisted radical resection of lung cancer (Da Vinci robot group) or thoracic surgery
4. The patient's cases were complete, and the statistics of various observation indexes were complete
5. The chief surgeon is a doctor in our department and has obtained the qualification of Da Vinci robot surgery.

The article "Application of Da Vinci Robot and Thoracoscopy in Radical Lung Cancer Surgery" was retracted in 2023. Reasons: unreliable results or conclusions; lack of ethics approval or compliance; concerns about the data; concerns about the peer review.

Case exclusion criteria were as follows:

1. Postoperative pathological report confirmed tuberculosis or other benign lesions
2. The TNM stage of lung cancer was stage IV
3. Traditional thoracotomy
4. The patient's case data were incomplete, and some observation indexes were missing
5. The chief surgeon is not qualified for the Da Vinci robot surgery.

### 3.2. Surgical Methods

#### 3.2.1. Da Vinci Robotic Surgery

*(1) The Incision*. A 12 mm small opening was made between the 7th rib of the axillary midline, an 8 mm small hole was cut between the 8th rib of the scapular line, the 5th rib between the axillary front line and the clavicular midline, and No. 1 and No. 2 operating arms were placed. Trocar was placed in the incision. The auxiliary operation port was 3 cm–4 cm between the 7th rib of the axillary midline. The assistant uses oval forceps to help the chief surgeon expose the operation part through the auxiliary hole. The surgeon in charge operates the Da Vinci manipulator. First, the doctor will loosen the lower pulmonary ligament and observe the development of pulmonary fissure and then decide to use anatomy or binomial surgery according to its development. The pulmonary vein, pulmonary artery, and bronchus are set free, and the cutting closure device is inserted from the auxiliary operation port by the assistant to nail and disconnect them, respectively. The hilar and mediastinal lymph nodes were routinely cleaned after smooth resection of the diseased lobes. After the operation, warm normal saline was poured into the chest, and the anesthesiologist was asked to ventilate the affected side of the lung. After checking that there was no air leakage at the bronchial stump, a closed thoracic drainage tube was placed.

#### 3.2.2. Thoracoscopic Surgery

The thoracoscopic group underwent three hole unidirectional thoracoscopic radical resection of lung cancer. The patient underwent double-lumen endotracheal intubation and contralateral one lung ventilation under general anesthesia. The healthy lateral position is taken, the body is tilted slightly forward, and different operation holes are taken according to the lung lobe where the lesion is located. During the operation, the assistant uses video-assisted oval forceps to help the main knife expose the operation space. The main knife doctor always dissects the lung root structure layer by layer in one direction with an ultrasonic knife or electrocoagulation hook, so as to minimize clamping and turning the lung lobes and prevent lung lobe injury. The pulmonary vein, bronchus, and pulmonary artery were cut and closed successively with an endoscopic cutting and closure device. After complete resection of the diseased lung lobe, the hilar and mediastinal lymph nodes were routinely cleaned.

The article "Application of Da Vinci Robot and Thoracoscopy in Radical Lung Cancer Surgery" was retracted in 2023. Reasons: unreliable results or conclusions; lack of ethics approval or compliance; concerns about the data; concerns about the peer review.

### 3.3. Observation Index

The observation indexes of the two groups of surgical cases included the number of lymph nodes cleaned during the operation, the amount of intraoperative bleeding, the operation time, the postoperative hospital stay, and the comfort of the surgeon.

### 3.4. Statistical Analysis

SPSS 18.0 software was used for statistical analysis. The pathological composition and TNM stage data were directly calculated by Fisher's exact probability method. Continuous variables were expressed as mean ± standard deviation (*x* ± *s*). The mean between groups was compared by *t*-test of two groups of independent samples, and *P* < 0.05 indicates the difference was statistically significant.

## 4. Experimental Result and Observations

### 4.1. Statistical Results of Clinical Data

#### 4.1.1. Statistical Results of Da Vinci Robot Group

As shown in Figure 3, this method can timely check the change position of lung cancer and achieve accurate positioning.

#### 4.1.2. Statistical Results of Thoracoscopy Group

Figure 4 shows the feature importance diagram. These 18 features are input into the “micro nonlinear” classifier to predict the final diagnosis results. The classifier consists of Table 1 penalized logistic regression model and a limit random tree model to fit the residuals of the linear model. An additional feature is that the output of Julian's mass detection model is used to predict the number of “abnormal masses” in patients' lungs.

As shown in Figure 5, in terms of data, doctors can establish a large sample single disease database to improve the quality of training data, standardize the labeling on this basis, form a high-quality training set, and learn to share and use data under laws and regulations. Doctors should also be the makers and executors of quality control and standards. For example, the standards of image acquisition and image quality are formulated, the expert consensus is formulated on the composition proportion, disease distribution, and lesion type of database construction, and the expert consensus is formed on the image signs and description of each single disease and the data marking of single disease AI model. A set of correct basic ethics is established to guide the design, management, and application of AI.

The article "Application of Da Vinci Robot and Thoracoscopy in Radical Lung Cancer Surgery" was retracted in 2023. Reasons: unreliable results or conclusions; lack of ethics approval or compliance; concerns about the data; concerns about the peer review.

## 5. Discussion

### 5.1. Feeling and Main Advantages of the Surgeon Operating the Da Vinci Robot

According to the operation feeling of the surgeon after the operation, the Da Vinci robot has many obvious advantages over thoracoscopy in the comfort of operation. First of all, the surgeon takes a sitting position during the operation. In the long-term complex operation, it can reduce the probability of making mistakes due to fatigue and increase the safety of the operation. Secondly, the joint of the Da Vinci robot surgical instrument can completely imitate the action of the human wrist, and the activity range of 7 degrees of freedom exceeds the 5 degrees of freedom of the human hand, which greatly improves the operation flexibility of surgery. Moreover, the machine has small operating instruments and high joint flexibility, which can be operated flexibly and freely in a narrow space. Compared with the Da Vinci robot, the operating instruments of thoracoscopy have less activity, and the joint flexibility is completely dependent on the manual adjustment of the chief surgeon so that the chief surgeon consumes more physical energy during the operation and is prone to wrist pain and fatigue. Finally, the endoscope of the Da Vinci robot is a high-resolution, three-dimensional lens with a magnification of more than 10 times for the surgical field, which can bring three-dimensional, high-definition images in the patient's body cavity to the chief surgeon, so that the chief surgeon has more advantages than ordinary video-assisted thoracoscopy in grasping the operating distance and identifying the anatomical structure. When the tissue structure is clearer, it is not easy to damage the structures such as the thoracic duct, recurrent laryngeal nerve, and tracheal membrane, so as to reduce postoperative complications such as chylothorax and vocal cord paralysis. The camera system controlled by the mechanical arm can provide a more stable field of vision than the video camera system manually supported by the thoracoscope, and it is easier to enter the deep cavity that is not easy to enter by the conventional endoscope. Moreover, Da Vinci robot radical lung cancer surgery only needs one assistant, while thoracoscopic radical lung cancer surgery needs two assistants, which can greatly reduce the labor cost. Finally, by integrating the computational technology, hand tremor can be filtered out, and eye-hand coordination can be realized. In such a stable operation environment, the operation is more accurate, the operation accidents are greatly reduced, the anatomical free tissue is clearer, and the satisfaction of the chief surgeon is greatly improved.

The article "Application of Da Vinci Robot and Thoracoscopy in Radical Lung Cancer Surgery" was retracted in 2023. Reasons: unreliable results or conclusions; lack of ethics approval or compliance; concerns about the data; concerns about the peer review.

### 5.2. Analysis of Statistical Results of Various Observation Indexes

There was no significant difference in gender, age distribution, pathological composition, and TNM stage between the two groups.

Through the experience of the chief surgeon, we can know that the mechanical operation arm of the Da Vinci robot is more flexible in the chest than the thoracoscopic instrument. The difficulty of lung cancer surgery is lymph node dissection. This may be related to the fact that the Da Vinci robot can clean more lymph nodes that are not easy to reach by thoracoscopy, and the cleaning is more thorough. In terms of the operation time, the value of the Da Vinci robot group was greater than that of the thoracoscopy group (*P* < 0.05). It shows that the operation time of the Da Vinci robot is longer than that of thoracoscopic surgery. This is mainly due to the short time for undergraduate Da Vinci robot surgery, less operating tables, and unskilled operation. In addition, the operation time such as the assembly of the Da Vinci robot arm is also calculated into the operation time.

With the increase of the Da Vinci robot surgery volume, the optimization of robot arm assembly process, and the improvement of surgical operation proficiency in the future, the operation time of the Da Vinci robot will also be reduced. At present, the cost of Da Vinci's surgery is high. Some patients are unwilling to choose Da Vinci's robotic surgery for economic reasons but choose thoracoscopic surgery with relatively low cost, resulting in less Da Vinci's robotic surgery than traditional thoracoscopic surgery.

In addition, there was no significant difference in intraoperative bleeding and postoperative hospital stay between the two groups (*P* > 0.05), indicating that the application of Da Vinci's robotic surgery system for radical lung cancer is as safe and effective as that of thoracoscopic radical lung cancer.

### 5.3. Da Vinci Robot System Needs to Be Improved

The first is the lack of force feedback. Surgeons can only rely on vision to distinguish the tissue but cannot distinguish the soft and hard degree of the tissue, which has no advantage in detecting the location of the mass. When clamping the tissue, it is easy to cause microvascular rupture and bleeding due to excessive force and affect the surgical field of vision. In addition, the mechanical operating arm of Da Vinci's robotic surgery system is too large, and the moving range and range are large during the surgical operation. In addition, the chief surgeon has no time to pay attention to the movement of the operating arm during operation, which is easy to make the operating arm accidentally hurt the assistant's head and cause physical injury to the assistant. In addition, the assembly of the Da Vinci robot manipulator is cumbersome and takes up a lot of valuable operation time. There is still a lot of room for improvement in how to improve the arm installation efficiency.

The article "Application of Da Vinci Robot and Thoracoscopy in Radical Lung Cancer Surgery" was retracted in 2023. Reasons: unreliable results or conclusions; lack of ethics approval or compliance; concerns about the data; concerns about the peer review.

At present, the cost of a single Da Vinci robot is high, and it cannot be equipped in all hospitals in the country. Moreover, the needle holder and gripper on its mechanical arm are consumables, which are used for a limited number of times and are expensive. The existence of these factors has led to its high operation cost. At present, many families in China are unable to bear such high operation costs, and there are few patients who choose the Da Vinci surgical system for radical resection of lung cancer, which makes it difficult to become a routine surgical method for all thoracic surgical diseases.

## 6. Conclusion and Future Directions

In this paper, we have explored the feasibility and safety of Da Vinci's robotic surgery system in the radical resection of lung cancer. All 22 patients in the Da Vinci robot group completed the operation under the Da Vinci robot operation system without conversion to thoracotomy. In the thoracoscopic group, 49 patients successfully completed the operation under thoracoscopy, and 2 patients were converted to thoracotomy. There was a significant difference between the two groups in the average operation time and the number of lymph nodes, but there was no significant difference in the amount of intraoperative bleeding and postoperative hospital stay. Compared with thoracoscopic radical lung cancer surgery, Da Vinci's robotic surgery system is equally safe and effective, and more lymph nodes are cleaned during surgery.

In the future, we are eager to expand the proposed model for other models and further enhance its safety and effectiveness.

## Figures and Tables

**Figure 1:** Da Vinci fourth generation equipment.

**Figure 2:** HD imaging display effect.

**Figure 3:** Detection effect.

**Figure 4:** Important features.

**Figure 5:** Test amplification effect.

**Table 1:** Comparison of clinical data between the Da Vinci robot and thoracoscopy (*X* ± *S*).

Clinical data	Robot group (*n* = 22)	Thoracoscopy group (*n* = 51)	*P* value
Age (years)	60.7±8.2	59.0±9.5	0.52
Operation time (min)	192.5±51.7	156.4±45.0	0.01
Intraoperative blood loss (ML)	175.0±79.6	202.0±112.1	0.38
Number of lymph nodes cleaned during operation	12.3±5.4	8.5±5.3	0.02
Postoperative hospital stay (days)	8.0±2.8	8.3±1.9	0.59

The article "Application of Da Vinci Robot and Thoracoscopy in Radical Lung Cancer Surgery" was retracted in 2023. Reasons: unreliable results or conclusions; lack of ethics approval or compliance; concerns about the data; concerns about the peer review.

## Data Availability

The datasets used and analyzed during the current study are available from the corresponding author upon reasonable request.
